# A RFID Authentication Protocol for Epidemic Prevention and Epidemic Emergency Management Systems

**DOI:** 10.1155/2021/1550993

**Published:** 2021-12-03

**Authors:** Xiuqing Chen, Xiao Zhang, Deqin Geng, Lei Zhou, Junshu Chen, Fan Lu

**Affiliations:** School of Medicine Information, Xuzhou Medical University, Xuzhou 221000, China

## Abstract

The outbreak of the novel coronavirus has exposed many problems in the auxiliary information system for epidemic prevention and control, which needs to be resolved by using methods such as the antitampering of logistics data and the management and control of epidemic materials. This article discusses the introduction of emerging technologies such as Radio Frequency Identification (RFID), which support privacy protection into the auxiliary information system for epidemic prevention and control. Recently, this paper found that Khwaja et al.'s protocol (RAPUS protocol) is susceptible to database impersonation attacks and reader impersonation attacks. Therefore, this article proposes the enhanced protocol, which not only perfectly solves the problems of the abovementioned protocols but also comprehensively compares multiple protocols. The enhanced protocol has higher efficiency and security. The security of the proposed protocol (RAPUS + protocol) is analyzed by GNY logic and the AVISPA model. The designed scheme can help realize the safety and traceability of epidemic prevention materials and improve the automation and decision-making efficiency of the epidemic prevention.

## 1. Introduction

Medical Internet of Things (IoMT) needs higher demand for security than the Internet of Things (IoT) when decreasing medical expense and enhancing the medical workpiece ratio. Khwaja et al.‘s protocol [1] uses symmetric cryptography to design a robust authentication protocol. In the enforcement of IoMT, RFID is required to create an identity authentication system as a key technology, which can effectually verify patients [2]. It is helpful to design a safe and efficient RFID for protecting user privacy, improving the safety of the IoMT system, and boosting the efficiency of medical staff to inspect and manage patients.

In medical scenes that need to efficiently verify a good deal of tags in a brief period, the employ of traditional per-tag protocols is inefficient and may put off the cure of patients. To solve the problem that uses the solution of homogeneous linear equations as a key to make the authentication data of the tag encipherment to further decrease the expense, Nikkhah et al. [3] proposed the LAPCHS protocol on account of the cloud healthcare system and analyzed and proved the safety of the protocol against various attacks by heuristic security analysis. Sarier et al. [4] proposed a new biometric based on nontransferable certificate scheme, which maintains the privacy and efficiency of biometric identification and can be easily integrated into the current BBIM system based on efficient brand and PS certificate.

Due to the low cost, high stability, and excellent characteristics of noncontact automatic identification of RFID system, it has been used in many fields, such as waste electronic product processing, farm management, and supply chain management [5–7]. In addition, in the field of healthcare, RFID technology is also widely used, such as drug management and vital signs detection [8, 9]. During the epidemic, RFID technology also participated in the establishment of the auxiliary information system for epidemic prevention, with the purpose of solving problems such as the management of epidemic material data and the management of epidemic information. Although the RFID system has many advantages in epidemic prevention and control, it faces the risks of security and privacy due to the usage of bottomed wireless media that enables (T, RE)'s mutual communication.

In order to design the secure RFID authentication solution, many protocols have been put forward to guarantee the security of RFID, but they have all been proved to have problems. In 2019, Khwaja et al. [1] proposed the lightweight authentication protocol. The authors claim that their protocol meets the necessary security requirements and solves most security issues. This paper finds that the protocol [1] is susceptible to database spoofing attacks, reader spoofing attacks, and asynchronous attacks. Therefore, this article proposes the new protocol on this basis, which can not only solve the problems of the abovementioned protocols but also can make the comprehensive comparison of multiple protocols, which has higher efficiency and security. The security of RAPUS + protocol is analyzed formally and informally through GNY logic, security verification tool AVISPA model. Through the above scheme, it is expected to improve the automation and decision-making efficiency of the epidemic prevention auxiliary information system.

This article analyzes the protocol [1] and improves realistic and lightweight certification protocol to guarantee protection against the known attacks:

1. The protocol [1] is susceptible to database impersonation attacks and reader impersonation attacks
2. The improved authentication protocols are proposed to resist all known attacks
3. RAPUS + protocol performs formal and informally security analysis and compares it with relevant existing protocols on security features and performance

## 2. Related Work

A variety of certification protocols have been put forward to protect RFID systems [10–22], especially for lightweight cryptographic primitives. But many schemes based merely on the lightweight primitives were verified to be insecure, as shown in Table 1.

In 2014, Cho et al. [10] put forward the hash-based protocol. Later, Safkhani et al. [11] pointed out that the protocol [10] cannot withstand DoS attacks and impersonation attacks. In the same year, the ECC-based RFID authentication protocols [12, 13] were proposed to ensure communication security in the medical environment and improve patient safety. However, Farash et al. [14] proved through analysis that the protocols [12, 13] cannot ensure forward secrecy. In 2015, Gope et al. [15] proposed the lightweight protocol. But Khwaja et al. [1] pointed out that their protocol is susceptible to collision, DoS attacks, and stolen attacks. In 2018, Fan et al. [16] proposed the ultralightweight LRMI protocol to protect medical privacy. However, Aghili et al. [17] analyzed that the LRMI protocol cannot withstand traceability attacks and simulation attacks and proposed the SecLAP protocol. However, under the analysis of Safkhani et al. [18], it is found that the protocol in [17] is susceptible to traceability attacks and asynchronous attacks. In the same year, Fan et al. [21] put forward the lightweight authentication scheme on the basis of quadratic. Later, Zhu et al. [22] analyzed and proved that their scheme is susceptible to forward secrecy and impersonation attacks. In 2019, Zhou et al. [19] put forward the protocol on the basis of secondary residues. But the protocol [20] cannot withstand asynchronous attacks. Naeem et al. [23] presented an RFID authentication protocol and suggested an improvement to cater to the correctness and scalability issues. Li et al. [24] presented a mutual-healing group key distribution scheme based on the blockchain which can effectively resist various attacks with small overhead on time and storage. Amin et al. [25] provided an effective solution to solve all existing problems regarding key protocol methods to enhance security. The AVISPA simulation results in the solution ensure that active and passive attacks are protected. Lin et al. [26] constructed a novel secure mutual authentication system and proved the security and privacy requirements, including anonymity, traceability, and confidentiality. Shahidinejad et al. [27] introduced a lightweight authentication protocol for IoT devices named Light-Edge using a three-layer scheme.

Section 3 reviews the protocol [1].  Section 4 demonstrates RAPUS + protocol. In Section 5, the security analysis of the RAPUS + protocol is checked.  Section 6 compares RAPUS + protocol with existing protocols. At last, Section 7 summarizes the article.

## 3. The Analysis of RAPUS Protocol

By examining the limitations of the RAPUS protocol, this section points out that it is susceptible to database impersonation attacks.  Table 2 demonstrates the symbols used in the RAPUS protocol.

The doctor and many patients make up every cluster. Patients are moved from one cluster to another. Via the DB Server, the registered patients are authenticated by the doctor and the cluster. The symmetric key *K*_*rs*_ is shared between each Doctor and DB. The improved authentication scheme is made up of two parts: the tag registration part and the tag certification part. We have the medical data through the protocol. Besides, we use the decentralization, traceability, and nontampering characters of blockchain technology to guarantee the security of data storage and sharing.

T registrations steps are as follows, as shown in Figure 1.

**Step 1 PTR 1.**

*ID*_*Ti*_ is submitted to the DB by each tag.

**Step 2 PTR 2.**

1. A random number *n*_*s*_ is generated by DB.
2. DB calculates *K*_*ts*_ = *h*(*ID*_*Ti*_||*n*_*s*_) ⊕ *ID*_*s*_.
3. DB randomly generates *r*_*i*_ and encrypts it with *s*_*x*_ to calculate one-time alias tag_*i*_'s identity *AID* = E_*sx*_(*ID*_*Ti*_||*r*_*Ti*_).
4. DB authenticates tag_*i*_ based on *AID*_*T*_.
5. DB stores and delivers *M*_2_ to tag.

**Step 3 PTR 3.**

Tag_*i*_ stores the information *M*_2_ = {*ID*_*Ti*_, *K*_*ts*_, *AID*} in its memory after receiving the messages from DB.

The registered *T* starts the certification procedure, which is presented in Figure 2. The specific steps are as follows:

Step PTA 1:
  1. Nt is generated by an RFID tag with IDTi.
  2. *N*_*x*_ = *K*_*ts*_ ⊕ *N*_*t*_ and *V*_1_ = *h*(*AID*_*Ti*_||*K*_*ts*_||*N*_*x*_||*R*_*i*_) are derived.
  3. T delivers *M*_A1_= {*AID*_*Ti*_,  *N*_*x*_,  *T*_1_, *V*_1_} to *R*_*i*_ to start the authentication request.
Step PTA 2:
  1. *R*_*i*_ of the *i*^*th*^ cluster verifies the timestamp freshness as (*T*_2_ − *T*_1_) ≤ ∆*T.*
  2. *N*_*r*_ is generated and *N*_*y*_ = *K*_*rs*_ ⊕ *N*_*r*_, *V*_2_ = *h*(*M*_A1_||*N*_*r*_||*K*_*rs*_) is calculated by *R*_*i*_.
  3. *R*_*i*_ delivers *M*_A2_={*N*_*y*_,  *R*_*i*_,  *V*_2_,  *M*_A1_, *T*_2_} to *S.*
Step PTA 3:
  1. *S* proves (*T*_3_−*T*_2_)≤∆*T* and then stems from *N*_*t*_ = *K*_*ts*_ ⊕ *N*_*x*_ and *N*_*r*_ = *K*_*rs*_ ⊕ *N*_*y*_.
  2. *V*_1_ = *h*(*AID*_*Ti*_||*K*_*ts*_||*N*_*x*_||*R*_*i*_) and *V*_2_ = *h*(*M*_*A*1_||*N*_*r*_||*K*_*rs*_) are calculated and verified by *S.*
  3. *S* decrypts *AID*_*Ti*_ as *D*_*Sx*_ (*ID*_*Ti*_||*r*_*i*_).
  4. After successful authentication, *S* calculates *V*_3_ = *h*(*R*_*i*_||*N*_*r*_||*K*_*rs*_) and *V*_4_ = *h*(*K*_*ts*_||*ID*_*Ti*_||*N*_*t*_).
  5. *AID*_*Ti*(*new*)_ = E_*Sx*_(*ID*_*Ti*_||*r*_*i*(*new*)_) is updated and *Z*_*T*_ = *AID*_*Ti*(*new*)_ ⊕ *K*_*ts*_ is computed by *S.*
  6. *S* delivers *M*_A3_= {*V*_3_,  *V*_4_, *ZT*, *T*_3_} to *R*_*i*._
Step PTA 4:
  1. *R*_*i*_ checks the freshness of the timestamp (*T*_4_−*T*_3_)≤∆*T.*
  2. *R*_*i*_ calculates h(*R*_*i*_||*N*_*r*_||*K*_*rs*_) and verifies its equality with the received *V*_3_.
  3. *R*_*i*_ delivers *M*_A4_= { *V*_4_,  *T*_4_,  *Z*_*T*_} to tag_*i*_.
Step PTA 5:
  1. Tag_*i*_ checks the freshness of the timestamp after receiving *M*_*A*4_.
  2. Tag_*i*_ calculates and renews *AID*_*Ti*(*new*)_=(*Z*_*T*_ ⊕ *K*_*ts*_), *AID*_*Ti*_ = *AID*_*Ti*(*new*)_, if Tag_*i*_ successfully verifies the messages (*T*_5_–*T*_4_) ≤ ∆*T*, *V*_4_*∗*? = *h*(*K*_*ts*_||*ID*_*Ti*_||*N*_*t*_).
  3. Tag_*i*_ saves the information.
  4. Otherwise, *AID*_*Ti*_ will not update.

### 3.1. Vulnerable to Database Impersonation Attacks for RAPUS Protocol

#### 3.1.1. Phase 1 (Learning)

After receiving *M*_A2_={*N*_*y*_, *R*_*i*_, *V*_2_, *M*_A1_, *T*_2_} from the reader, the DB performs as follows:

**STEP 1.1.**

*S* proves (*T*_3_−*T*_2_)≤∆*T* and then stems from *N*_*t*_=*K*_*ts*_ ⊕ *N*_*x*_ and  *N*_*r*_=*K*_*rs*_ ⊕ *N*_*y*_.

**STEP 1.2.**

*V*_1_=h(*AI*  *DT*  *i*‖*K*_*ts*_‖*N*_*x*_‖*R*_*i*_) and *V*_2_=h(*M*_A1_‖*N*_*r*_‖*K*_*rs*_‖*T*_2_) are calculated and verified by *S*.

**STEP 1.3.**

*S* decrypts *AI*  *DT*_*i*_ as D*S*_*x*_ (*I*  *DT*_*i*_*||r*_*i*_) in order to verify it.

**STEP 1.4.**

*V*_3_=h (*R*_*i*_‖*N*_*r*_‖*K*_*rs*_‖*T*_3_) and *V*_4_=h (*K*_*ts*_‖*I*  *DT*_*i*_‖*N*_*t*_‖*T*_3_) are calculated by *S*, after successful verification.

**STEP 1.5.**

*AI*  *DT*_*i* (*new*)_ =E*S*_*x*_ (*I*  *DT*_*i*_ ‖*r*_*i*(*new*)_) is updated and *Z*_*T*_=*AI*  *DT*  *i*_*new*_ ⊕ *KT*_*s*_ is computed by *S*.

**STEP 1.6.**

*S* delivers *M*_A3_ to *R*_*i*_.

#### 3.1.2. Phase 2 (Database Impersonation Attacks)

To imitate the database, the attacker starts a new session:

**STEP 2.1.**

The attacker eavesdrops *Z*_*T*_.

**STEP 2.2.**

The attacker maliciously modifies *Z*_*T*_′=*Z*_*T*_ ⊕ 1.

**STEP 2.3.**

The reader's verification method *V*_3_ does not check the integrity of *Z*_*T*_.

**STEP 2.4.**

At this time, the database impersonation attacks succeed.

### 3.2. Vulnerable to Reader Impersonation Attacks for RAPUS Protocol

#### 3.2.1. Phase 1 (Learning)

After receiving *M*_A3_={*V*_3_, *V*_4_, *Z*_*T*_, *T*_3_} from the DB, the reader performs the following steps.

**STEP 1.1.**

*R*_*i*_ checks freshness of the timestamp (*T*_4_−*T*_3_)≤∆*T*.

**STEP 1.2.**

*R*_*i*_ calculates h(*R*_*i*_‖*N*_*r*_‖*K*_*rs*_) and proves that it equals *V*_3_.

**STEP 1.3.**

*R*_*i*_ delivers *M*_A4_ to *tag*_*i*_.

#### 3.2.2. Phase 2 (Reader Imitation Attacks)

To imitate the reader, the attacker imitates the new routine:

**STEP 2.1.**

The reader continues to send the modified data *Z*_*T*_′(*Z*_*T*_ ⊕ 1) to *T*.

**STEP 2.2.**

T's validation method does not verify the integrity of *Z*_*T*_.

**STEP 2.3.**

The reader's impersonation attacks succeed.

### 3.3. Vulnerable to Asynchronous Attacks

**STEP 1.**

The above two processes lead to the wrong updating of cryptographic key *AID*'_*Ti*(*new*)_=(*Z′ T* ⊕ *K*_*Ts*_).

**STEP 2.**

In the second round of conversation, *T* key *AID*'_*Ti*(*new*)_ and *T* key *AID*_*Ti*(*new*)_=(*Z*_*T*_ ⊕ *K*_*Ts*_) stored in the database are inconsistent.

**STEP 3.**

Therefore, it results in asynchronous attacks.

## 4. The Improved RAPUS + Protocol

RAPUS + protocol is shown in Figure 3.

Step PTA 1:
  1. *N*_*t*_ is generated by RFID tag with *ID*_*Ti*_.
  2. *N*_*x*_ = *K*_*ts*_ ⊕ *N*_*t*_ and *V*_1_ = *h*(*AID*_*Ti*_||*K*_*ts*_||*N*_*x*_||*R*_*i*_) are exported.
  3. T delivers *M*_A1_={*AID*_*Ti*_,  *N*_*x*_,  *T*_1_,  *V*_1_} to *R*_*i*_.
Step PTA 2:
  1. *R*_*i*_ of the *i*^*th*^ cluster first proves the timestamp freshness as (*T*_2_−*T*_1_)≤∆*T*, as soon as the request is received from *T*.
  2. *N*_*r*_ is generated by *R*_*i*_.
  3. *N*_*y*_ = *K*_*rs*_ ⊕ *N*_*r*_ and *V*_2_ = *h*(*M*_*A*1_||*N*_*r*_||*K*_*rs*_||*T*_2_) are computed.
  4. *R*_*i*_ delivers *M*_A2_={*N*_*y*_,  *R*_*i*_,  *V*_2_,  *M*_A1_,  *T*_2_} to *S.*
Step PTA 3:
  1. *S* proves (*T*_3_−*T*_2_) ≤∆*T* and then stems from *N*_*t*_ = *K*_*ts*_ ⊕ *N*_*x*_ and *N*_*r*_ = *K*_*rs*_ ⊕ *N*_*y*_.
  2. *S* calculates and proves *V*_1_ = *h*(*AID*_*Ti*_||*K*_*ts*_||*N*_*x*_||*R*_*i*_) and *V*_2_ = *h*(*M*_*A*1_||*N*_*r*_||*K*_*rs*_||*T*_2_).
  3. *S* decrypts *AID*_*Ti*_ as *D*_*Sx*_(*ID*_*Ti*_||*r*_*i*_) to verify it.
  4. After verifying successfully, *S* renews *V*_3_ = *h*(*R*_*i*_||*N*_*r*_||*K*_*rs*_||*Z*_*T*_) and *V*_4_ = *h*(*K*_*ts*_||*ID*_*Ti*_||*N*_*t*_||*Z*_*T*_).
  5. *AID*_*Ti*(*new*)_ = E_*Sx*_(*ID*_*Ti*_||*r*_*i*(*new*)_) is updated and *Z*_*T*_ = *AID*_*Ti*(*new*)_ ⊕ *K*_*ts*_ is computed by *S.*
  6. *S* delivers *M*_A3_={*V*_3_,  *V*_4_,  *Z*_*T*_,  *T*_3_} to *R*_*i*_.
Step PTA 4:
  1. *R*_*i*_ verifies the freshness of the timestamp (*T*_4_−*T*_3_)≤∆*T* after receiving *M*_A3_.
  2. *R*_*i*_ calculates and verifies h(*R*_*i*_ ||*N*_*r*_ ||*K*_*rs*_ ||*Z*_*T*_) = *V*_3_.
  3. *R*_*i*_ delivers *M*_A4_={*V*_4_,  *T*_4_,  *Z*_*T*_} to tag_*i*_ after successful verification.
  4. If not, *R*_*i*_ ends the session.
Step PTA 5:
  1. Tag_*i*_ checks the freshness of the timestamp after receiving *M*_A4._
  2. Tag_*i*_ calculates and renews *AID*_*Ti*(*new*)_=(*Z*_*T*_ ⊕ *K*_*ts*_), *AID*_*Ti*_ = *AID*_*Ti*(*new*)_ if Tag_*i*_ verifies the message *V*_4_*∗*? = *h*(*K*_*ts*_*||ID*_*Ti*_*||N*_*t*_*||Z*_*T*_).
  3. Tag_*i*_ saves the information.
  4. Otherwise, *AID*_*Ti*_ will not update.

## 5. The Analysis of RAPUS + Protocol

The security of the RAPUS + protocol is analyzed through formal analysis and explains the informal security features under the GNY logic model and AVISPA model.

### 5.1. The Informal Analysis

In the following subsections, we analyze the security of the RFID system.

#### 5.1.1. Mutual Authentication between Tag and Server

The DB verifies *AID*_*Ti*_ and *V*_1_ = *h*(*AID*_*Ti*_||*K*_*ts*_||*N*_*x*_||*R*_*i*_) in *M*_1_ to authenticate RFID tag. Only the legitimate *T* can form the effective request *M*_1_, which includes the two parameters. As effective *AID*_*Ti*_, it only knows legal T. Besides, the legal tag only knows (*ID*_*T*_, *K*_*ts*_). The RFID tag can use *V*_4_ and *M*_3_ in *M*_4_ to authenticate the legitimacy of the DB. The mutual authentication property can be achieved by RAPUS + protocol.

#### 5.1.2. Anonymity

The most basic element of the secure protocol is anonymity. The personal information of the user is protected by a secure scheme so that the adversary has no access to any information. The protocol has achieved strong anonymity. During the registration part, the RFID tag used *M* = {*ID*_*Ti*_, *K*_*ts*_, *AID*} to identify the *S* through RFID-Reader.

The messages *M*_*A*1_ = {*AID*_*Ti*_, *N*_*x*_, *V*_1_, *T*_1_} have been delivered to the *S* through a public channel in the authentication part. The adversary cannot attain the identity of the RFID tag even if the adversary gets the message *M*_1_ for the reason that *AID*_*Ti*_ is the one-time alias identity of T. The initial identity is kept encoded in *AID*_*Ti*_. It can only be encoded by the DB using *K*_*ts*_. Therefore, the adversary cannot destroy the RFID tag's authentic identity. In this way, we achieve the anonymity of the protocol.

#### 5.1.3. Traceability

A safe protocol can protect any identity information of the participants from illegal users. The traceability of the RFID tag may be caused by identifying information. RAPUS + protocol cannot reveal the login information of the conversation that causes the security attack.

The protocol needs to use (*N*_*t*_, *N*_*r*_, *r*_*i*_). It is impossible for the adversary to achieve any random number in the RFID system because the RFID tag's new one-time alias identity *AID*_*Ti*_ has already been used. Therefore, the protocol meets the untraceability.

#### 5.1.4. Backward/Forward Secrecy

It is essential for security protocols to ensure that the information transferred during a phase is not threatened and traced by the adversary, as it may generate defects in the certification phase between *T* and *S*. In our proposed scheme, the previous and next sessions will not be affected, even if the identity *ID*_*T*_ is lost. The encrypted *AID*_*Ti*_ is updated in each new session to ensure it. Therefore, the backward and forward secrecy of the RAPUS + protocol can be guaranteed.

#### 5.1.5. Scalability

In RAPUS + protocol, the detailed procedure is used to verify if any *T* is not performed by the RFID Server *S*. Oppositely, *S* disposes *AID*_*Ti*_ to verify *T* and makes a quick response to T. Therefore, RAPUS + protocol gets more stable.

#### 5.1.6. DoS Attacks

For any random key which is in charge of verification or authentication of *T*, the protocol is not based on them. Instead, it is on the basis of *AID*_*Ti*_. Moreover, it is well encoded and renewed for each transaction. Hence, the proposed scheme defenses against DoS attack.

#### 5.1.7. Replay Attacks

In the replay attack, to authenticate S, the attacker may postpone and repeat the transferred information. (T, RE, DB) are included in RAPUS + protocol. For authentication, {*M*_1_, *M*_2_, *M*_3_, *M*_4_} are exchanged through the public channel. Accessible to the messages, the attackers try to launch the replay attacks.

Nevertheless, due to the messages delivered with the fresh timestamp *T*, the attempt will fail. The adversary request will be repulsed each time in the event of timestamp's ineffectiveness. Besides, the adversary cannot launch the attacks if it cannot calculate the parameters of the messages, because all messages' parameters are updated by the participants for every new session. RAPUS + protocol is able to resist replay attacks.

#### 5.1.8. Location Tracking Attacks

The authentic identity of the RFID tag is not delivered firsthand. Therefore, it has been delivered in the encoded form for authentication between the RFID tag and S. And only the server can decrypt through its secret key. Besides, in every new session, the unpredictability of messages is continually renewed. Therefore, the adversary cannot seek out the location. Any attempt to find the location will finally become a failure.

#### 5.1.9. Impersonation Attacks

To authenticate the server, adversary *A* holds up the messages of the valid *T* and changes it. On this occasion, adversary *A* needs to issue the legitimate message request including (*N*_*y*_, *R*_*i*_, *V*_2_, *M*_*A*1_, *AID*_*Ti*_). In order to achieve it, *AID*_*Ti*_ is encrypted and calculated and cannot be forged by adversary *A*.

Besides, to submit the legitimate request for certification as the valid *T*, adversary *A* demands various other timestamps and parameters too. Adversary *A* is impossible to know the real parameters used for certification. Therefore, it has no ability to verify its validity as *T* to the DB. RAPUS + protocol for RFID system can resist any forgery attack reluctantly.

#### 5.1.10. Stolen-Verifier Attacks

All the validation and verification keys are encrypted and stored in the DB. Although the data and keys are both stolen from the DB, they cannot be decrypted and extracted by adversary *A*. Moreover, the original data saved in DB cannot be altered or modified by adversary *A*. Therefore, the RAPUS + protocol resists the stolen-verifier attacks.

### 5.2. The Formal Analysis Using GNY Logic

In order to guard against major attacks, the proposal of the security protocol design must be analyzed ahead of execution. The fundamental assumptions are presented in Table 3.

The aims verified by RAPUS + protocol are as follows:

- Goal 1: *R*_*i*_ | ≡ $tag\overset{AID_{T}}{⟷}R_{i}$
- Goal 2: *R*_*i*_| ≡ *T*| ≡ $tag\overset{AID_{T}}{⟷}R_{i}$
- Goal 3: *S*_*j*_ | ≡ $R_{i}\overset{AID_{T}}{⟷}S_{j}$
- Goal 4: *Sj* | ≡ *R*_*i*_| ≡ $R_{i}\overset{AID_{T}}{⟷}S_{j}$
- Goal 5: *R*_*i*_ | ≡ $S_{j}\overset{AID_{T}}{⟷}R_{i}$
- Goal 6: *R*_*i*_| ≡ *S*_*j*_ | ≡ $S_{j}\overset{AID_{T}}{⟷}R_{i}$
- Goal 7: *T*| ≡ $R_{i}\overset{AID_{T}}{⟷}tag$
- Goal 8: *T*| ≡ *R*_*i*_ | ≡ $R_{i}\overset{AID_{T}}{⟷}tag$

The protocol messages generated by the parser are as follows:

- *M*_1_*: T ⟶R*_*i*_*: AID*_*T*_*, N*_*x*_*:< N*_*t*_*>K*_*ts*_*, V*_1_*, T*_1_
- *M*_2_*: R*_*i*_*⟶S*_*j*_*: M*_1_*, N*_*y*_*:< N*_*r*_*>K*_*rs*_*, R*_*i*_*, V*_2_*, T*_2_
- *M*_3_*: S*_*j*_*⟶R*_*i*_*: V*_3_*, V*_4_*, Z*_*t*_*:<AID*_*Ti*_*>∗*_*Kts*_*, T*_3_
- *M*_4_*: R*_*i*_*⟶ T: V*_4_*, T*_4_*, Z*_*t*_*:< AID*_*Ti*_*>*_*Kts*_

The goals (*G*_1_, *G*_2_, *G*_3_, *G*_4_, *G*_5_, *G*_6_, *G*_7_, *G*_8_, *G*_9_) are made to verify the RAPUS + protocol that has been certified. The sequence of logical assumptions is employed in the parser export to achieve the security goals by considering the various assumptions.

In *M*_1_, *T*_1_ is the timestamp of *T*. Using the seeing rule, we can get

(1) $$\begin{array}{c} R_{i}⊲AIDT_{i},SID,N_{x}:<N_{t}{>}_{Kts},T1. \end{array}$$

Applying the message-meaning rule and the previous step result,

(2) $$\begin{array}{c} \;R_{i}\left|\equiv tag\right|∼N_{t}. \end{array}$$

Using the freshness-conjuncatenation rule and the previous step results,

(3) $$\begin{array}{c} R_{i}\left|\equiv tag\right|\equiv N_{t} \end{array}$$

According to the jurisdiction rule and the previous step result,

(4) $$\begin{array}{c} R_{i}|\equiv N_{t}. \end{array}$$

Applying the previous step result and the session-key rule,

(5) $$\begin{array}{c} R_{i}|\equiv tag\overset{{AID}_{Ti}}{⟷}R_{i}\left(Goal1\right). \end{array}$$

Using the nonce-verification rule,

(6) $$\begin{array}{c} R_{i}\left|\equiv tag\right|\equiv tag\overset{{AID}_{Ti}}{⟷}R_{i}\left(Goal2\right). \end{array}$$

In *M*_2_, *T*_2_ is the timestamp of *R*_*i*_. Applying the seeing rule, we get

(7) $$\begin{array}{c} S_{j}⊲M1,N_{y}:<N_{r}>K_{rs},T2,V2. \end{array}$$

According to the message-meaning rule and the previous step result,

(8) $$\begin{array}{c} S_{j}\;\left|\equiv R_{i}\right|∼N_{r}. \end{array}$$

By the freshness-conjuncatenation rule and the previous step result, we get

(9) $$\begin{array}{c} \;S_{j}\;\left|\equiv R_{i}\right|\equiv N_{r}. \end{array}$$

Through the jurisdiction rule and the previous step result,

(10) $$\begin{array}{c} S_{j}\;|\equiv N_{r}. \end{array}$$

Applying the S_10_ and the *SK* rule,

(11) $$\begin{array}{c} S_{j}\;|\equiv R_{i}\overset{{AID}_{Ti}}{⟷}S_{j}\left(Goal3\right). \end{array}$$

According to the nonce-verification rule and the previous step result,

(12) $$\begin{array}{c} S_{j}\;\left|\equiv R_{i}\right|\equiv R_{i}\overset{{AID}_{Ti}}{⟷}\;S_{j}\left(Goal4\right). \end{array}$$

In *M*_3_, *T*_3_ is the timestamp of *S*_*j*_. Through the seeing rule, we get

(13) $$\begin{array}{c} R_{i}⊲V3,V4,Z_{t}<AIDT_{inew}{>}_{K_{ts}}^{*},T3. \end{array}$$

Applying the message-meaning rule and S_13_,

(14) $$\begin{array}{c} R_{i}\;\left|\equiv S_{j}\right|∼AIDT_{inew}. \end{array}$$

Through S_14_ and the freshness-conjuncatenation rule,

(15) $$\begin{array}{c} R_{i}\;\left|\equiv S_{j}\right|\equiv AIDT_{inew}. \end{array}$$

According to the assumption S_15_ and jurisdiction rule,

(16) $$\begin{array}{c} R_{i}\;|\equiv AIDT_{inew}. \end{array}$$

Applying S_16_ and the session-key rule,

(17) $$\begin{array}{c} R_{i}\;|\equiv S_{j}\overset{{AID}_{inew}}{⟷}R_{i}\left(Goal5\right). \end{array}$$

Using the nonce-verification rule,

(18) $$\begin{array}{c} R_{i}\;\left|\equiv S_{j\;}\right|\equiv S_{j}\overset{{AID}_{inew}}{⟷}R_{i}\left(Goal6\right). \end{array}$$

In *M*_4_, *T*_4_ is the timestamp of *R*_*i*_. Applying the seeing rule,

(19) $$\begin{array}{c} tag⊲V4,Zt<AIDT_{inew}\geq {>}_{ts},T4. \end{array}$$

Through the message-meaning rule and S_19_,

(20) $$\begin{array}{c} tag\;|\equiv R_{i}\;|∼AIDT_{inew}^{'}. \end{array}$$

According to S_20_ and the freshness-conjuncatenation rule,

(21) $$\begin{array}{c} tag\;\left|\equiv R_{i}\right|\equiv AIDT_{inew}. \end{array}$$

Applying the jurisdiction rule and S_21_,

(22) $$\begin{array}{c} \;tag|\equiv AIDT_{inew}. \end{array}$$

By the session-key rule, we get

(23) $$\begin{array}{c} \;tag|\equiv R_{i}\overset{{AID}_{inew}}{⟷}tag\left(Goal7\right). \end{array}$$

Finally, according to the nonce-verification rule,

(24) $$\begin{array}{c} tag\left|\equiv R_{i}\right|\equiv R_{i}\overset{{AID}_{inew}}{⟷}tag\left(Goal8\right). \end{array}$$

As a result, it is proved that (*T*, *R*_*i*_, *S*_*j*_) achieve successful reciprocal certification and obtain the session-key agreement safely.

### 5.3. The Protocol Verification Using AVISPA Tool

The AVISPA is the formal security protocol analysis tool. It uses the High-Level Protocol Specification Language (HLPSL) to specify the sequence of messages exchanged among different entities. The basic role is the module consisting of the action of each entity. The entities combine multiple basic roles into the composed role to interact with each other. The analyzed protocol's security goals are specified in the goal phase. It has four back ends, including OFMC, CL-Atse, SATMC, and TA4sp, which use different kinds of techniques to show whether the RAPUS + protocol is safe or not. The tool supplies tracking of the steps that lead to the attack and uses the Dolev-Yao intruder model that can eavesdrop, intercept messages, modify passing traffic, or insert bogus data. In our proposed scheme, we describe different entities' actions by defining the basic role and how the entities in the composed role interact with each other. The results present that our proposed scheme is “safe” against OFMC with regard to the security goal in Figure 4. Appendix A shows all source programs by AVISPA.

### 5.4. Performance Analysis and Comparison

This phase conducts the comparative analysis between the RAPUS + protocol and the existing protocol. First of all, we compare the existing protocol with the RAPUS + protocol in terms of security requirements. Besides, based on the calculation cost, we compare the RAPUS + protocol with the existing protocol. Lastly, we compare the RAPUS + protocol with existing protocols in regard to model analysis.

#### 5.4.1. Security Requirements

This section analyzes the existing authentication protocols based on symmetric keys from the perspective of security requirements.  Table 4 presents the comparisons between the proposed agreement and the existing agreement [1, 10, 15, 28–30].

Table 4 shows the insecurities of existing protocols [1, 10, 15, 28–30]. The result shows that only RAPUS + protocol can provide all the above security features, such as mutual authentication, untraceability, anonymity, the backward/forward secrecy, scalability, collision attacks, DoS attacks, replay attacks, location tracking attacks, stolen-verifier attacks, database impersonation attacks, and reader impersonation attacks.

#### 5.4.2. Computational Cost

The computation cost analysis of existing related protocols [1, 10, 15, 28–30] with RAPUS + protocol is given in this section.  Table 5 presents the analysis of computation cost.

In the protocol proposed in [15], the computational cost of each (*T*, *R*, *S*) is 5*Th*, 2*Th*, and 7*Th*, so the total cost is 14*Th*. The protocol proposed in [29] needs 2*Th*, 2*Th*, and 3*Th* for each (T, *R*, S), and the total cost is 7*Th*. The cost of protocol demonstrated in [30] is 4*Th*, 2*Th*, and 6*Th* correspondingly, amounting to 12*Th*. In the protocol proposed in [10], each (*T*, *R*, *S*) generates 3*Th*, 2*Th,* and 5*Th* cost correspondingly, so the total cost is 10*Th*. The cost of protocol demonstrated in [28] is 2*Th*, 3*Th*, and 5*Th* correspondingly, amounting to 10*Th*. The protocol proposed in [1] needs 2*Th*, 2*Th*, and 4*Th* +2*Tse* for each (*T*, *R*, *S*), so the total cost is 8*Th* + 2*Tse*. In comparison, *T* requires 2*Th*, the reader requires 1*Th*, and the server requires 3*Th* + 2*Tse*, and the total cost is 6*Th* + 2*Tse* in the protocol proposed in this article. In general, the protocol proposed in this article has a relatively smaller computation cost and is the only one that can withstand all known attacks.

### 5.5. Comparisons of Model Analysis

This section describes a model analysis of RAPUS + protocol with existing multitag authentication protocols in Table 6.

The results show that most protocols lack or have no model analysis. In the proposed authentication protocol, the secrecy attacks are analyzed by automatic cryptographic protocol verifier tools AVISPA. GNY logic is applied to verify the reciprocal certification.

## 6. Conclusion

The auxiliary information system for epidemic prevention and control has integrated traditional medical systems with RFID technology. However, the antitampering of logistics data and management and control of epidemic materials are still challenges. In this article, we prove that the RAPUS protocol is susceptible to database impersonation attacks, reader impersonation attacks, and asynchronous attacks. Then, the RAPUS + protocol is proposed. The security analysis of the RAPUS + protocol has been conducted through GNY logic, AVISPA model. Additionally, the comparisons of RAPUS + protocol with the existing protocols prove the superiority in security, computational cost, and model analysis. Based on RAPUS + protocol, the safety and management of epidemic prevention materials will be greatly improved.

## Figures and Tables

**Figure 1:** Tags registration phase.

**Figure 2:** Tags authentication phase.

**Figure 3:** The improved RAPUS + protocol.

**Figure 4:** AVISPA execution of RAPUS + protocol.

**Table 1:** The issues of lightweight authentication protocols.

Lightweight authentication protocols	Security issues
Cho et al. [10]	DoS and impersonation attacks [11]
Zhao et al. [12], Zhang et al. [13]	Cannot ensure forward secrecy [14]
Gope and Hwang [15]	Collision, DoS, and stolen-verifier attacks [1]
Fan et al. [16]	Traceability attacks and simulation attacks [17]
Aghili et al. [17]	Traceability attacks and asynchronous attacks [18]
Fan et al. [21]	Forward secrecy and impersonation attacks [22]
Zhou et al. [19]	Asynchronous attacks [20]

**Table 2:** Symbols and definitions of the RAPUS protocol.

Symbols	Definitions
*T*; *S*; *R*	RFID tag; database (DB); reader device
*ID*_*Ti*_; *AID*_*Ti*_; *SID*; *R*_*j*_; *N*_*t*_; *N*_*r*_	*i* ^th^ tag identity; one-time tag alias identity; shadow identity
*K*_*ts*_; *K*_*emg*_	*j* ^th^ reader identity; Tag random number; reader random number
*Tr*_*seq*_; *K*_*rs*_	Shared key (shared emergency key) of server and tag
*r*_*j*_	Track sequence number (used by both *S* and *T*)
*h*(.); ⊕; ||	Hash function; the exclusive XOR operation; concatenation

**Table 3:** The assumptions used for RAPUS + protocol under the GNY logic.

*T*_*i*_ {*ID*_*Ti*_}	*Reader* {*R*_*i*_}	*Database Server* {*S*_*j*_}
*T*| ≡ #(*N*_*t*_)	*R*_*i*_ | ≡ #(*N*_*r*_)	*S*_*j*_ | ≡ #(*AID*_*Ti*_) (*r*_*i*_)
*T*| ≡ *S*_*j*_ ⇒ *r*_*i*_	*R*_*i*_ | ≡ *S*_*j*_ ⇒ *r*_*i*_	*Sj* | ≡ *R*_*i*_ ⇒ *N*_*r*_
*T*| ≡ *R*_*i*_ ⇒ *N*_*r*_	*R*_*i*_ | ≡ *T* ⇒ *N*_*t*_	*Sj* | ≡ *T* ⇒ *N*_*t*_

**Table 4:** Security requirements comparisons.

Requirements	[27]	[23]	[28]	[29]	[30]	[10]	[15]	[1]	Ours
SR1	√	√	×	×	×	√	×	√	√
SR2	√	√	×	×	×	√	--	--	√
SR3	√	√	×	×	×	√	--	--	√
SR4	√	√	√	×	×	√	--	--	√
SR5	√	√	×	×	×	√	--	--	√
SR6	√	√	×	×	×	×	×	√	√
SR7	√	√	×	×	×	×	×	√	√
SR8	√	√	×	×	×	×	√	√	√
SR9	--	--	--	--	--	--	--	--	√
SR10	--	--	--	--	--	--	--	--	√
SR11	--	--	--	--	--	--	--	×	√
SR12	--	--	--	--	--	--	--	×	√

SR1: mutual authentication. SR2: tag untraceability. SR3: tag anonymity. SR4: backward/forward secrecy. SR5: scalability. SR6: collision attacks. SR7: DoS attacks. SR8: replay attacks. SR9: location tracking attack. SR10: stolen-verifier attacks. SR11: database impersonation attacks. SR12: reader impersonation attacks.√: yes provides; ×: does not provide.

**Table 5:** Comparisons of computation cost.

Computation cost	[15]	[29]	[30]	[10]	[28]	[1]	Ours
^CC^tag	5*T*_*h*_	2*T*_*h*_	4*T*_*h*_	3*T*_*h*_	2*T*_*h*_	2*T*_*h*_	2*T*_*h*_
CC_Ri_	2*T*_*h*_	2*T*_*h*_	2*T*_*h*_	2*T*_*h*_	3*T*_*h*_	2*T*_*h*_	1*T*_*h*_
CC_S_	7*T*_*h*_	3*T*_*h*_	6*T*_*h*_	5*T*_*h*_	5*T*_*h*_	4*T*_*h*_ + 2T_se_	3*T*_*h*_ + 2T_se_
^CC^Total	14*T*_*h*_	7*T*_*h*_	12*T*_*h*_	10*T*_*h*_	10*T*_*h*_	8*T*_*h*_ + 2T_se_	6*T*_*h*_ + 2T_se_

CC: computation cost; *T*_*h*_: CC of single hash function; *T*_se_: CC of symmetric encryption/decryption.

**Table 6:** Comparisons of model analysis.

Formal model	[27]	[23]	[28]	[29]	[30]	[10]	[15]	[1]	Ours
BAN	×	×	×	×	×	×	×	×	×
GNY	×	×	×	×	×	√	×	×	√
AVI	√	×	×	×	×	×	×	×	√
ProVerif	×	×	×	×	×	√	×	×	×

## Data Availability

The data served to support the findings of this study are contained within the article.

## Appendix

### A. The Source Programs under AVISPA Model

  role reader(
   R,T,S:agent,
   H:hash_func,
   SND_TR,RCV_TR,SND_SR,RCV_SR:channel(dy)
  )
  played_by R
  def = 
     local
    State:nat,
    R0,DID,C0,RID,C1,R1,
    C2,Tid,C3,TID,OID,C4,
    C5,C6,TS1,TS3,C7,SR,C8,KRC,C9,
    Tidnew,C10,C11,C12:text
  const
  tag_reader_c3,tag_reader_c7,reader_tag_c7:protocol_id
  init State: = 0
  transition
(1) State = 0/\RCV_SR(start) = |>
   State': = 1
   /\R0': = new()
   /\C0':=H(R0'.DID)
   /\C1': = xor(DID,RID)
   /\SND_TR(R0'.C0'.C1′)
(2) State = 1/\RCV_TR(C2'.C3'.C4'.C5'.C6'.R1′) = |>
   State': = 2
   /\C7': = xor(C3′,xor(H(RID.DID),TS1))
   /\C8': = xor(OID,SR)
   /\SND_SR(TS1.C7'.C8'.H(RID).H(TS1.C7'.C8'.H(RID).KRC).R1′)
   /\witness(R,T,reader_tag_c7,C7′)
(3) State = 2/\RCV_SR(C9'.H(C9'.KRC)) = |>
   State': = 3
   /\Tidnew': = xor(R1,Tid)
   /\C10': = xor(Tidnew',SR)
   /\SND_SR(C10'.TS3.H(C10'.TS3.KRC))
(4) State = 3/\RCV_SR(C11'.H(C11′,KRC)) = |>
   State': = 4
   /\C12': = xor(H(TID.DID.OID),R1)
   /\SND_TR(C12′)
  end role
  role tag(
   R,T,S:agent,
  H:hash_func,
   SND_RT,RCV_RT:channel(dy)
  )
  played_by T
  def = 
     local
    State:nat,
    R0,DID,C0,RID,C1,R1,
    C2,Tid,C3,TID,OID,C4,
    C5,C6,TS1,TS3,C7,SR,C8,KRC,C9,
    Tidnew,C10,C11,C12:text
  const tag_reader_c3,tag_reader_c7,reader_tag_c7:protocol_id
  init State: = 0
  transition
(1) State = 0/\RCV_RT(R0'.C0'.C1′) = |>
   State': = 1
   /\R1': = new()
   /\C2': = xor(RID,xor(Tid,R1′))
   /\C3': = xor(DID,xor(H(TID.DID.R1′),RID))
   /\C4': = xor(OID,H(RID.R0′))
   /\C5':=H(OID.R0'.C3′)
   /\C6':=H(RID.R0'.R1′)
   /\SND_RT(C2'.C3'.C4'.C5'.C6'.R1′)
   /\witness(T,R,tag_reader_c3,C3′)
   /\witness(T,R,tag_reader_c5,C5′)
(1) State = 1/\RCV_RT(C12′) = |>
   State': = 2
  end role
  role server(
   R,T,S:agent,
   H:hash_func, SND_RS,RCV_RS:channel(dy)
  )
  played_by S
  def = 
     local
    State:nat,
    R0,DID,C0,RID,C1,R1,
    C2,Tid,C3,TID,OID,C4,
    C5,C6,TS1,TS3,C7,SR,C8,KRC,C9,
    Tidnew,C10,C11,C12:text
  const tag_reader_c3,tag_reader_c7,reader_tag_c7:protocol_id
  init State: = 0
  transition
(1) State = 0/\RCV_RS(TS1.C7'.C8'.H(RID).H(TS1.C7'.C8'.H(RID).KRC).R1′) = |>
  State': = 1
  /\C9': = xor(Tid,SR)
  /\SND_RS(C9'.H(C9'.KRC))
(2 ) State = 1/\RCV_RS(C10'.TS3.H(C10'.TS3.KRC)) = |>
  State': = 2
  /\Tidnew': = xor(C10′,SR)
  /\C11': = xor(H(TID.DID.OID),xor(Tidnew',SR))
  /\SND_RS(C11'.H(C11′,KRC))
  end role
  role session(
   R,T,S:agent,
    H:hash_func
    )
   def = 
    local
      SSR,RSR,STR,RTR,SRT,RRT,SRS,RRS:channel(dy)
    composition
  reader(R,T,S,H,STR,RTR,SSR,RSR)
    /\tag(R,T,S,H,SRT,RRT)
    /\server(R,T,S,H,SRS,RRS)
  end role
  role environment()
    def = 
    const
      r,t,s:agent,
      h:hash_func,
      tag_reader_c3,tag_reader_c7,reader_tag_c7:protocol_id
    intruder_knowledge = {r,t,s}
  composition
    session(r,t,s,h)
    /\session(r,t,s,h)
    /\session(r,t,s,h)
  end role
  goal
  authentication_on tag_reader_c3
  authentication_on tag_reader_c7
  authentication_on reader_tag_c7
  end goal
  environment()
